RETRACTED

# Investigation of the Role of *Leuconostoc mesenteroides* subsp. cremoris in Periodontitis around Abutments of Fixed Prostheses

**DOI:** 10.1155/2022/8790096

**Published:** 2022-05-20

**Authors:** Saif Ali Mohammed Hussein, Rehab Aamer Kareem, Ali Maki Hamed Al-Dahbi, Mequanint Birhan

**Affiliations:** ^1^Department of Medical Laboratory Technique, Dijlah University College, Iraq; ^2^Department of Prosthodontics, College of Dentistry, University of Dijlah, Iraq; ^3^Dentistry Department, Dijlah University College, Iraq; ^4^Department of Mechanical Engineering, Mizan-Tepi University, Ethiopia

## Abstract

This study included the role of *Leuconostoc mesenteroides* subsp. cremoris in oral diseases such as periodontitis. *Material and Method*. Isolation and identification of *Leuconostoc mesenteroides* subsp. cremoris from a saliva sample of twenty patients wearing fixed dental prostheses suffering from periodontitis followed by estimating susceptibility generally to the most common antibiotics and specifically to chlorhexidine (CHX) to determine the MIC of CHX and also screening of the strength of biofilm production under aerobic and anaerobic conditions; here, the study included six groups: Group I: screening of biofilm formation under aerobic condition, Group II: screening the MIC of CHX effect on biofilm formation under aerobic condition, Group III: screening of the MIC of CHX effect on preformed biofilm under aerobic condition, Group IV: screening of biofilm formation under anaerobic condition, Group V: screening of MIC of CHX effect on biofilm formation under anaerobic condition, and Group VI: screening of MIC of CHX effect on preformed biofilm under anaerobic condition. *Results*. The results showed that about 5 (25%) isolates were identified as *L. mesenteroides* subsp. cremoris, while 75% are other isolates. Furthermore, susceptibility results to antibiotic showed the sensitivity to penicillin (100%), azithromycin (100%), ciprofloxacin (100%), tetracycline (100%), gentamicin (100%), doxycycline (100%), vancomycin (100%), ofloxacin (60%), chloramphenicol (80%), ampicillin (80%), and cefoxitin (60%). On the other side, the biofilm production assays revealed that all isolates were moderate biofilm former under the aerobic and anaerobic conditions but for the biofilm treated with MIC of CHX, the current study noticed that the strength of the biofilm became weaker in aerobic and anaerobic conditions; regardless, the strength of the biofilm under anaerobic conditions was higher than in that under aerobic conditions, with no significant differences at *p* ≤ 0.05 depending on the statistical analysis (*T*-test) before and after the treatment with MIC of CHX in aerobic and anaerobic conditions. *Conclusions*. The presence of *mesenteroides* subsp. cremoris in the oral cavity is due to eating foods and vegetables; based on the strength of the biofilm and sensitivity tests, the isolates have less pathogenicity in the oral cavity due to the weakness of the biofilm production and the lack of resistance to antibiotics.

RETRACTED

## 1. Introduction

Probiotics are live nonpathogenic microorganisms that are provided to the host to enhance microbial community balance [1]. The use of microbiome treatment in oral cavity homeostasis is a relatively recent notion, as a viable alternative to antibiotics in the treatment of a variety of oral disorders such as periodontitis and dental caries. The mode of mechanism action can be characterized as direct or indirect. For the effect in direct mode, the probiotic organisms have an effect on pathogenic organism itself [2].

The indirect route of action involves probiotic microbes regulating the host's response to infections [2]. Some researches focused on *Leuconostoc mesenteroides* subsp. mesenteroides as a viable probiotic. Furthermore, this microorganism has important technological properties, such as the ability to produce acetaldehyde, dextran, acetoin, and diacetyl; also, proteolytic enzymes and lipolytic enzymes at the same time have the ability to grow under extremely stressful conditions [3].

Many *L. mesenteroides* species generate a variety of organic acids, as well as a class of antibacterial chemicals known as bacteriocins (such as carnosin and leuconocin). These chemical substances inhibit both gram-negative and gram-positive bacteria [4]; few studies have found that employing Leuconostoc as a probiotic strain has a high potential. [5] demonstrated that the use of Leuconostoc as a probiotic strain was superior to the probiotic Lactobacillus strain currently in clinical use in generating cytokines [6].

Furthermore, it has been found that *L. mesenteroides* can prevent pathogen growth and can be employed as a safe probiotic for further research [7, 8]. L. mesenteroides has shown significant antibacterial activity against gram-positive and gram-negative bacteria [9] like *S. pyogenes* [10] and *G. anatis* [11].

## 2. Material and Method

### 2.1. Sample Collection

A total of 20 specimens (saliva) were collected from fixed dental prosthesis patients complaining from periodontal diseases and suspended in 1 ml phosphate buffer saline (PBS) then transported to the microbiology and immunology laboratory in Dijla University.

### 2.2. Isolation and Identification of Bacteria

Approximately 100 *μ*l of samples was inoculated into MRS agar plates for 24 hr in 37°C; the isolates were characterized by cultural and morphological features [12] and Vitek 2 system.

RETRACTED

### 2.3. Antimicrobial Susceptibility

Antibiotic susceptibility testing will be carried out using a modified Kirby-Bauer Disk diffusion method and commercially available antibiotic discs. The size of the inhibitory zone was used to classify stains as susceptible, intermediately resistant, or resistant, according to the manufacturer's instructions; this corresponded to the WHO's interpretation criteria: penicillin (P, 10 g), azithromycin (AZM, 15 g), ciprofloxacin (CIP, 5 g), tetracycline (T, 30 g), gentamicin (G, 10 g), doxycycline (DO, 30 g), vancomycin (VA, 30 g), ofloxacin (OF, 5 g), chloramphenicol (C, 30 g), and ampicillin (A, 10 g).

### 2.4. CHX Susceptibility Test

Agar diffusion method was followed as described in [CLSI, 2016]. The isolates were adjusted to1.5 × 10^∗8^CFU/ml and cultured on Mueller-Hinton agar-containing wells (6 mm in diameter). 0.1 ml of chlorhexidine gluconate 2% *w*/*v* was added into the wells, then incubated under aerobic condition; the same steps were repeated under anaerobic conditions (GasPak Jar) for 24 hr at 37°C.

### 2.5. Estimation of Minimum Inhibitory Concentration (MIC) of CHX

The inoculums were adjusted to roughly 1.5 × 10∗8 CFU/ml, and 1 ml was transferred to tubes containing 1 ml of MIC. The tubes were incubated at 37°C for 24 hours, and the quantity of growth in the tubes containing CHX was matched to the growth-control tubes (no CHX) as the control. The organism's development in the tubes was impeded, as seen with the naked eye [13].

### 2.6. Screening the Biofilm Formation

This assay included six groups as shown in Table 1.

### 2.7. Screening of Biofilm Production in Bacterial Isolates under Aerobic and Anaerobic Condition

In the procedure described by O'Toole [14], 24 hr old isolates were inoculated in tryptic soy broth and incubated for 18 hours at 37°C in, then diluted 1 : 100 with fresh tryptic soy broth; then, wells of plates (96-well flat-bottom tissue culture plates) were loaded with 0.2 ml of the diluted bacteria and with only broth media (without bacteria) serving as a control (blank) to verify sterility; the following formula was used to determine the biofilm formation strength:

1. OD ≤ ODC = nonbiofilm former (NBF)
2. ODC < OD ≤ 2X ODC = weak biofilm former (WBF)
3. 2 XC < OD ≤ 4 XC = moderate biofilm former (MBF)
4. OD > 4X ODC = strong biofilm former (SBF)

OD stands for optical density and ODC stands for optical density of control.

### 2.8. Screening Effect MIC of CHX on Biofilm Production under Aerobic and Anaerobic Condition

This assay was performed according to Tanner et al. [15] and modified. 200 *μ*l of the particular antibiotic (MIC of CHX) dilution in tryptic soy broth was put into the wells (96-well plate); then, the isolates were diluted with 0.2 ml fresh tryptic soy broth; subsequently, 200 *μ*l of the suspension was loaded into the wells and the other wells were loaded only with broth (without bacteria) serving as control (blank) to check sterility followed by incubation at 37°C for 24 hr; the following formula was used to determine the biofilm formation strength:

1. OD ≤ ODC = nonbiofilm former (NBF)
2. ODC < OD ≤ 2X ODC = weak biofilm former (WBF)
3. 2 XC < OD ≤ 4 XC = moderate biofilm former (MBF)
4. OD > 4X ODC = strong biofilm former

OD stands for optical density and ODC stands for optical density of control.

RETRACTED

### 2.9. Screening Effect of MIC of CHX on Performed Biofilm under Aerobic and Anaerobic Condition

Isolates of 24 hr old were diluted to 0.2 ml of tryptic soy broth followed by 100 *μ*l loaded into the wells of plate; after the incubation period at 37°C for 24 hr for biofilm formation, the medium was removed gently, the generated biofilm was then rinsed three times with PBS to eliminate nonadherent cells, and at that time, 200 *μ*l of MIC of CHX was added and then, the plate was incubated at 37°C for 24 hr; this test was renewed in the absence of MIC of CHX as a control [15], and the biofilm production strength was calculated as follows:

1. OD ≤ ODC = nonbiofilm former (NBF)
2. ODC < OD ≤ 2X ODC = weak biofilm former (WBF)
3. 2 XC < OD ≤ 4 XC = moderate biofilm former (MBF)
4. OD > 4X ODC = strong biofilm former

OD stands for optical density and ODC stands for optical density of control.

### 2.10. Statistical Analysis

The statistical analysis was achieved by *T*-test probability ≤ 0.05.

## 3. Results and Discussion

A total of 20 samples were collected from patients with gradient collected; approximately 5 (25%) *L. mesenteroides* isolates were identified according to morphological and Vitek system beside 75% of other isolates in Figure 1.

These findings agreed with [16, 17], which identified *S. salivarius*, S. anginosus, *L. mesenteroides*, and *L. sakei* (through morphological and genetic analysis from dental caries patients, However, the presence of these bacteria may be ascribed to food residues in the mouth in persons who have been diagnosed with acute severe caries. According to Ananieva et al. [18], both *L. sakei* and *L. mesenteroides* have been proven in some studies to be environmentally sustainable agents against foodborne pathogens in the mouth [19].

The isolates showed sensitivity to penicillin (100%), azithromycin (100%), ciprofloxacin (100%), tetracycline (100%), gentamicin (100%), doxycycline (100%), vancomycin (100%), ofloxacin (60%), chloramphenicol (80%), ampicillin (80%), and cefoxitin (60%) (see Figure 2).

RETRACTED

The findings of the current study agreed with [20] during the study of Leuconostoc sp. from acute cellulitis and acute apical periodontitis showing. Among the 93 exudate samples, 2 (1.6%) were positive for Leuconostoc spp. that have been isolated from one acute facial cellulitis and an acute apical periodontitis. Leuconostoc isolates showed 100% sensitivity to lincosamides (lincomycin and clindamycin). The beta-lactam antibiotics to which isolates were 100% sensitive are piperacillin, tobramycin, amoxicillin-clavulanic acid, gentamycin, piperacillin-tazobactam, and penicillin G. By contrast, isolates were 100% resistant to trimethoprim-sulfamethoxazole. Sensitivity was 50% for macrolides (spiramycin and erythromycin) and for the 3rd-generation cephalosporin antibiotics (cefotaxime, cefuroxime, cefixime, and ceftriaxone).

Anyways, the dental surgeons currently use broad-spectrum antibiotics. In most cases, the prescription of antibiotics in endodontic infections is empirical and an overuse is observed [21]. This contributes to the emergence of antibiotic-resistant bacterial strains [22]. The study reported in this work is about the isolate. Unlike many gram-positive bacteria, Leuconostoc species commonly demonstrate high-level resistance to vancomycin, with preserved sensitivity to most other antibacterial agents [23]. Furthermore MIC of CHX for isolates was ≤3.5 (*μ*g/ml) depending on the inhibition zones, under aerobic conditions and under anaerobic conditions in the inhibition zone (7.5 ± 0.06,7 ± 0.46), respectively; however, CHX's antibacterial activity caused the bacterial cytoplasmic membrane being damaged. However, resistance to CHX was attributed to the alterations in the cell membrane [24].

Moreover, *L. mesenteroides* isolates were moderate biofilm former (MBF) under aerobic and anaerobic conditions (Table 2). But when the biofilm was treated by MIC of CHX, that noticed the biofilm became weaker under aerobic and anaerobic conditions; however, in the anaerobic conditions, the strength of the biofilm formation was higher than that in aerobic condition; the statistical analysis in the *t*-test has no significant difference between the aerobic and anaerobic conditions after and before the treatment by CHX (Table 3).

Leathers and Bischoff [25] revealed that *L. citreum* and *L. mesenteroides* produce glucans that are comparable to commercial dextran; however, these strains differed significantly in their ability to build biofilms. Biofilm density was found in these strains. As a result, biofilm-forming capability differed greatly between strains in both species, and the kinds of polysaccharides generated did not appear to have an effect on biofilm formation.

RETRACTED

However, CHX has lower effectiveness against the formed biofilm after 24 hr due to the biofilm previously developed by isolates as known by the bacterial biofilm used by bacteria to avoid drugs, ingestion by phagocytosis, and other antimicrobial agents [26, 27], but the activity of antibiotic CHX showed more against preformed biofilm formation attributed to the antimicrobial action against free bacterial isolates and no biofilm formed yet [28].

Regardless, the CHX showed to be less effective under anaerobic condition against biofilm formation and performed biofilm. Leuconostoc is a lactic acid bacterium that produced biofilms [29]. A prior study found that when L. mesenteroides was incubated in a high CO_2_ environment, the exudate volume and dextran quantity were much larger than when incubated in an aerated environment. The overexpression of the dextransucrase-encoding genes dsrD and dsrT in *L. mesenteroides* during the first 4 to 8 hours of exposure to high CO_2_ levels relative to aerated conditions is linked to dextran synthesis [30, 31].

*L. mesenteroides* subsp. has important technological properties and ability to grow under stress conditions [3], although few research studies have observed the probiotic characteristics of this bacterium [32, 33].

On the other hand, various studies isolated L. mesenteroides from the oral cavity [18]; recently, different studies [19, 34] reported that *L. mesenteroides* biofilm has an important role as an antibacterial, including the oral bacteria as Streptococcus mutans in which dextran-producing Leuconostoc strains are capable to inhibit S. mutans biofilm formation [35]. Ahmaed and Awad [34] revealed that the biofilm produced by *L. mesenteroides* showed antimicrobial activity; *Staphylococcus aureus*, Salmonella spp., *Escherichia coli*, Klebsiella spp., *Pseudomonas aeruginosa*, *Streptococcus mutans* that appear to have *L. mesenteroides* can produce exopolysaccharides especially soluble dextran [36]. Many Leuconostoc mesenteroides species produce many organic acids in addition to a group of antimicrobial compounds, especially protein products called bacteriocines and like bacteriocines (such as carnosin and leuconocin). This compound inhibited gram-negative and gram-positive bacteria by damaging the cell or protein synthesis and nucleic acid [4].

## 4. Conclusion

Based on the results of this study, the existence of *L*. mesenteroides subsp. cremoris, in the oral cavity is due to eating foods and vegetables; based on the strength of the biofilm and sensitivity tests, the isolates have less pathogenicity in the oral cavity due to the weakness of the biofilm production and the lack of resistance to antibiotics; finally, these isolates are more active under anaerobic conditions.

RETRACTED

## Figures and Tables

**Figure 1:** Percentage occurrence of *L. mesenteroides* in 20 patients suffering from periodontitis.

**Figure 2:** Susceptibility of *L. mesenteroides* forward antibiotics.

**Table 1:** 

Groups	Biofilm formation methods
Group I	Screening of biofilm formation under aerobic condition
Group II	Screening of MIC of CHX effect on biofilm formation under aerobic condition
Group III	Screening of MIC of CHX effect performed biofilm under aerobic condition
Group IV	Screening of biofilm formation under anaerobic condition
Group V	Screening of MIC of CHX effect biofilm formation under anaerobic condition
Group VI	Screening of MIC of CHX effect performed biofilm under anaerobic condition

**Table 2:** Biofilm formation and effect of CHX toward the biofilm formation under aerobic and anaerobic condition.

Biofilm groups	Mean	S.D	S.E
Group 1	0.123	0.029	0.021
Group II	0.114	0.007	0.005
Group III	0.103	0.009	0.011
Group IV	0.240	0.130	0.092
Group V	0.170	0.087	0.062
Group VI	0.261	0.230	0.012

**Table 3:** Paired sample test (*T*-test).

Paired groups	Mean	*T*	Sig.
Group I-Group II	0.008	0.321	0.802
Group IV-Group V	0.0700	2.333	0.258
Group 1-Group IV	-0.117-	-1.035-	0.489
Group II-Group V	-0.055-	-0.982-	0.506
Group III–Group VI	-0.035-	-0.882-	0.406

## Data Availability

The data underlying the results presented in the study are available within the manuscript.
